The article "Construction Method of Industrial College in Vocational Colleges Based on Cluster Analysis Algorithm" was retracted in 2023. Reasons: unreliable results or conclusions; lack of ethics approval or compliance; concerns about the data; concerns about the peer review.

# Construction Method of Industrial College in Vocational Colleges Based on Cluster Analysis Algorithm

**DOI:** 10.1155/2022/3278395

**Published:** 2022-06-13

**Authors:** Xiaorong Liu

**Affiliations:** Wuxi Vocational College of Science and Technology, Wuxi, 214028 Jiangsu, China

## Abstract

In the context of the combination of industry and education, the construction of industrial colleges in vocational colleges can drive the scientific development of specialty settings in colleges and universities, and promote the way for colleges to expand students' practical teaching under the teaching of theoretical knowledge, and it is also an effective way for students to stimulate their learning enthusiasm and innovation enthusiasm. Colleges and universities can increase the direction and characteristics of specialist settings in colleges while enhancing instructors' professional level through school-business collaboration, and growing measures of talent training in colleges and universities plays a significant guiding role. The way to set up industrial colleges in vocational colleges reflects the development characteristics of talent training mode in the new era, and it is also an effective way to meet the practical training of students and the actual needs of society. It is a new school running mode of transforming productivity, cooperation, and mutual benefit, which is very worthy of promotion and development. This paper analyzes the problems existing in the construction of industrial colleges in vocational colleges in China and finds out the corresponding solutions. A path method of industrial college construction in vocational colleges based on the cluster analysis algorithm is proposed. The validity of this model is verified by experiments, which lays a foundation for the construction of industrial colleges in vocational colleges.

## 1. Introduction

For vocational colleges, the main purpose of training students is to shoulder the actual tasks in the actual work and be able to take the lead in the production, operation, and each job with professional knowledge, rich experience, and skilled technology [1]. The biggest difference between vocational education and ordinary higher education is that the talents trained belong to applied skilled talents, that is, they can combine professional knowledge with the practical operation. On the one hand, they complete the study of theoretical knowledge during school study; on the other hand, they complete the study, production, and service under the training mode of school-enterprise cooperation [2]. The college of the industry provides a practical and innovative platform for the majority of higher vocational students so that they can have a real simulated operation environment before they formally take up their jobs.

The way of talent training in vocational colleges is to face the market and serve the industry. Only when the talent training meets the actual needs of the current society and industry for talents can the effective development of individual talents be realized, and the teaching direction is suitable for post-application. Over the years, the development of vocational education in China has made continuous reform and innovation with the continuous transformation of the industrial structure, but it is still difficult to meet the actual needs of the market. The construction of industrial colleges in vocational colleges aims at the needs of enterprises and trains students. It is very necessary for students to adapt to industry standards in advance while cultivating professional knowledge [3]. This can not only improve the fit between the professional setting of vocational colleges and the industrial structure but also enable colleges to recognize the shortcomings of professional courses with the assistance of the industrial college, which plays a great role in promoting the professional setting of colleges and market research [4]. At present, most of the industrial colleges of vocational colleges in China are carried out in the way of school-enterprise cooperation, in which enterprises provide venues, equipment, and technology, and colleges provide teaching venues and teaching teacher management content. This cooperation mode takes advantage of each other in terms of the management system, teacher team or training base construction has a strong educational purpose, and can develop strengths and avoid weaknesses at the same time [5]. The respective advantages of enterprises and colleges are reflected in the construction of industrial colleges, so as to realize the win-win strategy of education and production. For vocational colleges, it can not only have better practical significance in the overall professional setting and skill improvement but also play a great role in promoting the cultivation of double qualified education and enhancing the core competitiveness of the college [6]. The construction path of industrial colleges in vocational colleges is shown in Figure 1.

The industrial college of vocational colleges is neither a university nor a college of education in the traditional sense, but rather a learning organization that refers to the collaboration between schools and businesses to develop talent. It aims to provide college students with a high-quality and high-skilled learning system and strives to transform students' professional theoretical knowledge into practical operation ability. At present, China's higher vocational industrial colleges generally set up special venues in the college and build them in the form of joint secondary colleges with relevant enterprises in the industry, so as to provide students with practice places and create a practice platform [7]. Industry university cooperation is a new mode of contemporary vocational education. Under this mode, it provides a good development opportunity for the construction of industrial college of vocational colleges. However, it is undeniable that the institutional setting and management mode of enterprises and colleges are completely different [8]. The continuous development and prosperity of this educational mode also stimulate some contradictions in the system, institution, and management of the industrial college. If these contradictions are not solved, it is bound to restrict the daily management of the Institute of Technology to a great extent and seriously hinder the further deepening of school-enterprise cooperation.

The following is the paper's organization paragraph: Section 2 discusses the related work. The design of the application model is examined in Section 3. The experiments and results are discussed in Section 4. Finally, the research job is completed in Section 5.

## 2. Related Work

In this section, we explain the development status of industrial colleges in vocational colleges, research status of construction path of industrial college, and research status of clustering algorithm in detail.

### 2.1. Development Status of Industrial Colleges in Vocational Colleges

The school running mode of school-enterprise cooperation is an effective carrier for the development of colleges and enterprises. It is not only a way for enterprises to cultivate talents but also a teaching measure for vocational colleges to actively set up professional industries [9]. The two sides can realize cooperation on the basis of mutual benefit and establish vocational colleges as a training base for professional and skilled talents. However, in terms of the current construction mode of industrial colleges in most vocational colleges, the school-enterprise cooperation is too unitary in form and content, taking the order type talent training and post-practice mode as the primary mode of cooperation, and the lack of deeper cooperation mode limits the way of industry education integration and talent transmission, which is not conducive to giving full play to the role of talent training base in vocational colleges [10]. The development status of the Institute of Technology is shown in Figure 2.

The main body of the construction of industrial college is implemented by the cooperation between enterprises and colleges. However, due to the great differences in the organization and management methods of both sides, the lack of a detailed management scheme and supervision system in the management of the industrial college is very disadvantageous from the perspective of enterprises or colleges. Enterprises cannot integrate into the management of industrial colleges, and colleges and universities cannot play a real educational role [11]. In the process of cooperation, there is a lack of detailed rules for the implementation of cooperation schemes, resulting in unclear rights and responsibilities and uneven distribution of interests, which is very likely to lead to the lack of implementation power of cooperation subjects, which fundamentally hinders the development of school-enterprise cooperation [12]. As the main mode of school-enterprise cooperation in vocational colleges at the present stage, the entrusted training order training mode will still have various teaching problems due to the immaturity of the educational mechanism, such as students' academic performance, behavior performance, implementation countermeasures, internship, and employment [13]. It is similar to the phenomenon of signing an employment agreement while ignoring academic performance and school behavior. Both students and parents believe that an employment agreement can ensure students' future employment, which has brought great trouble to vocational colleges in daily teaching management.

### 2.2. Research Status of Construction Path of Industrial College

The construction of mixed ownership industrial colleges in vocational colleges should be in line with the coordinated development of regional industrial clusters and the improvement of educational quality and the optimization of professional structure in vocational colleges [14]. It should not only accomplish scientific rationality of the best combination of industrial and educational elements but also achieve rapid resource structure and efficiency growth [15]. At the same time, we can achieve in-depth integration of talent training mode, curriculum system construction, teaching method reform, scientific research innovation, teacher team construction, and so on between industrial enterprises and vocational colleges through mutual integration and derivation between industrial layout and related majors. To build a mixed ownership industrial college in vocational colleges, we must first clarify the essential attributes, main characteristics, and school running orientation of the mixed ownership industrial college, and scientifically understand the differences between the mixed ownership industrial college and the secondary college [16]. A secondary college is a secondary teaching unit attached to a higher vocational college. It is different from a mixed ownership industrial college in terms of property right structure, school running subject, founding purpose, and operating mechanism.

In addition, the establishment of a variety of industrial clusters and research institutes, as well as the close integration of various industrial clusters and industrial associations that hinder the sustainable development of the park, should break through the bottleneck of the main body of the park and the integration of multiple industries, institutions, and research institutes, as well as the close cooperation between the two sides [17], the development model of interoperability and mutual progress. The establishment of corporate identity is fundamental for the mixed ownership industrial college to settle down. At present, under the legal system and framework of higher education in China, the legal person status of mixed ownership vocational colleges cannot be relied on, and the legal person status of mixed ownership industrial colleges is more difficult to determine. Vocational colleges are not-for-profit legal persons. Mixed ownership industrial colleges undertake the main function of public welfare vocational education [18]. It is obviously inappropriate to be positioned as for-profit legal persons; the participation of nonpublic capital such as industrial capital and private capital in running schools inevitably requires capital appreciation, which is not in line with the characteristics of nonprofit legal persons. Therefore, the mixed ownership industrial college can be positioned as a special legal person. As an independent educational and teaching institution, the college of mixed ownership industry is not for profit [19]. It is engaged in public welfare vocational education, technology development, social services, and other functions. It is jointly funded and established with industrial enterprises, social organizations, and individuals, which is in line with the basic characteristics of special legal persons [20].

Therefore, the legal person status of mixed ownership industrial college must be clarified by special laws and regulations or clear provisions. Many existing education policy documents encourage the development of industrial colleges with mixed ownership characteristics. Only by issuing special policy documents on the legal personality of the college of mixed ownership industry can we clarify the legal personality of the college of mixed ownership industry from the legal level [21]. Due to the diversification of school running subjects, the mixed ownership industrial college should follow the dual development principles of market law and education law. Improving the management mechanism and building a modern governance structure is not only an important guarantee for the efficient operation of the industrial college but also a prerequisite for realizing the goal of talent training [22]. Second, we should effectively participate in the management of the mixed ownership industrial college as stakeholders. The construction path of the industrial college is shown in Figure 3.

### 2.3. Research Status of Clustering Algorithm

The standard NMF method's single nonnegative constraint beam cannot suit the needs of many fields; hence, there are still certain flaws and restrictions. Researchers develop a neighbor network and a weighted adjacency matrix based on the similarity between data points in order to mine the possible manifold structural information between high-dimensional data and suggest the graph's regular nonnegative matrix decomposition [23]. Considering that a single cluster center in NMF and GNMF is not enough to describe the complex structure of the original data, researchers use multiple center points to represent the category of samples, so as to propose the local center structure nonnegative matrix decomposition [24].

In order to adaptively learn the local manifold structure, the researchers propose the concept of adaptive neighborhood and adaptively assign neighbors to each data point, so as to propose a non-negative matrix decomposition with the adaptive domain. Generally speaking, the cluster center is surrounded by some points with low local density, and these points are far away from other high-density points [25]. Then, the researchers proposed the density peak algorithm, which calculates the distance of the nearest neighbor and arranges it according to the density to obtain multiple peak points of the data, so as to obtain the clustering center to realize the efficient clustering of the data [26]. However, the nearest neighbor graph constructed by GNMF is based on the traditional Euclidean distance, which sometimes cannot accurately describe the real distance between samples when dealing with complex data structures [27]. Furthermore, while the LCSNFM model stipulates the same number of centers for each cluster, the architecture of various clusters varies in practice. This description is obviously flawed [28].

Although the LCSNFM algorithm uses multiple center points to represent the sample points in a cluster, the structure of each cluster is different in practical application. It is obviously unreasonable to specify the same number of center points for different clusters, and the optimal clustering results cannot be obtained for the data with complex structures [29]. To solve this problem, this paper proposes PNMF. The density peak algorithm is used to locate numerous density peak points for the data set, and then the linear combination of density peak points is used to create cluster center points for clustering. The regular term is also integrated into the NMF framework [30], and the geodesic distance is used to generate the manifold nearest neighbor graph.

## 3. Design of Application Model

### 3.1. Basic Principle of Clustering Algorithm

The algorithm finds multiple density peak points of the data, constructs a bipartite graph with its peak points and sample points, constructs a data nearest neighbor graph based on geodesic distance, and integrates it into the nonnegative matrix decomposition model. Clustering is the process of grouping items into distinct classes or clusters based on their features and particular rules, with the goal of making data within each class as similar as feasible while data between classes is as dissimilar as possible. The general steps of clustering are shown in Figure 4.

Therefore, for the selection of density peak points, the local density of sample points and the distance from the density center are comprehensively considered. In practical application, the number of samples in different classes varies greatly, and the density is also different, which will lead to the uneven distribution of the selected peak points. Take all sample points as a candidate set of density peak points, then assess each sample point's local density and distance from the density center, and choose a sample point in order from large too small. The similarity measurement step is used to measure the similarity of different data in the same feature space.

Firstly, the local density of each sample point is calculated, and multiple density peaks are found from the data set by using the local density. It specifies multiple center points for each cluster and constructs a bipartite graph by using the density peak points and sample points. In addition, the geodesic distance under manifold structure is used to construct the nearest neighbor graph of data, so as to describe the local geometric relationship and make the distance between sample points more accurate. In order to prove the effectiveness of the algorithm, this paper compares the clustering effect of the algorithm on several facial data sets, and text and sound data sets. Experimental results show that PNMF has better clustering performance than other NMF algorithms. The clustering performance of GN-MF and NMFAN based on the Euclidean distance nearest neighbor graph is not as good as that of PNMF based on the manifold distance nearest neighbor graph, which shows that the traditional Euclidean distance cannot well and accurately show the true distance between data in the face of more complex and high-dimensional data. Because of the limits of its cluster center selection, LCSNMF is less effective than PNMF, while standard NMF clustering performs poorly due to a lack of constraints. The nonnegative matrix decomposition model is a common data dimensionality reduction method. In the research of existing nonnegative matrix decomposition algorithms for clustering, each category is generally represented by one or more designated central points.

The clustering algorithm based on the partition is to divide the data into *k* classes, and *K* should be less than the total number of data. The division method needs to know the number of clusters in advance, randomly select the initial cluster center, and the other objects will be divided into which class near the cluster center. Then, an objective function is optimized to iteratively find a new cluster center, and the remaining objects are classified until the cluster center is no longer changed or the number of iterations is reached. The partition-based clustering algorithm iterates continuously according to the optimization evaluation function, which is simple to calculate. It is suitable for large-scale data sets and spherical clusters. However, the number of clusters should be determined in advance and sensitive to the initial clustering center. The obtained solution is not necessarily the global optimal solution but maybe the local optimal solution. The probability that each data point is selected as the cluster center shall meet the following mathematical expression.

(1) $$\begin{array}{c} P_{i}=\frac{D{\left(x_{i}\right)}^{2}}{\sum_{i=1}^{n}\;D{\left(x_{i}\right)}^{2}}. \end{array}$$

If the structure of the data set is unknown, we need to use internal measurement methods. To quantify clustering quality, we usually utilize the intracluster variance, which is the sum of squares of intracluster errors. Its mathematical expression is as follows.

(2) $$\begin{array}{c} V\left(C\right)=\underset{C_{k}\in C}{\sum }\;\underset{i\in C_{k}}{\sum }\;d{\left(i,\mu_{k}\right)}^{2}. \end{array}$$

The effectiveness index is the linear combination of the average dispersion of clusters and the overall separation between clusters, which is defined as the following expression.

(3) $$\begin{array}{c} \text{SD}\left(\text{C}\right)=\alpha \text{Scat}\left(\text{C}\right)+\text{Dis}\left(C\right). \end{array}$$

At present, most clustering algorithms need to customize some parameters, and the selection of these parameters directly affects the final clustering effect. Therefore, the influence of these parameters should be considered when selecting the clustering quality measurement method. At the same time, these measurement standards can also help us set the parameter values. When choosing clustering quality evaluation methods, we should also consider the structure of the data itself. At present, there is no measurement method suitable for all application fields. We choose the appropriate measurement method according to the specific situation. When clustering data objects, we need to evaluate the difference between objects, that is, the commonly known distance. Among them, the Euclidean distance function is the most commonly used measurement method, and its expression is as follows.

(4) $$\begin{array}{c} d\left(i,j\right)={\left[\overset{n}{\underset{k=1}{\sum }}\;{\left(x_{ik}-x_{jk}\right)}^{2}\right]}^{1/2}. \end{array}$$

In traditional clustering methods, each attribute of the object is treated equally, and their contribution to clustering is equal. However, in practical application, the internal properties of objects are different, and the importance of each attribute will be different.

### 3.2. Improved Clustering Algorithm

At present, the most popular fuzzy clustering algorithm is the fuzzy mean algorithm. Its goal is to minimize the criterion function and gradually obtain a more accurate membership matrix. It is easy to fall into the local optimal solution of the iterative center selection process. The goal of the FCM algorithm is to find the optimal prototype matrix and the corresponding membership matrix to minimize the objective function given by the following formula.

(5) $$\begin{array}{c} J=\overset{C}{\underset{i=1}{\sum }}\;\overset{N}{\underset{j=1}{\sum }}\;{\left(u_{ij}\right)}^{m}d_{ij}^{2}. \end{array}$$

The parameter *d*_*ij*_ is obtained from the following formula:

(6) $$\begin{array}{c} d_{ij}=||s_{j}-\beta_{i}||. \end{array}$$

After calculating the membership of all objects, you can calculate the new cluster prototype. When the prototype stabilizes, the process stops. In other words, the prototype generated in the previous iteration is very close to the prototype. In order to adjust the performance of particle swarm optimization and local search ability of particle swarm optimization in the search process, a simple and effective inertia weight adjustment strategy is introduced into the particle swarm optimization algorithm. The new function is as follows:

(7) $$\begin{array}{c} \omega_{l}\left(t\right)=\left(\ln\left(2.1+t\right)\right)\wedge \left(-z\right). \end{array}$$

New velocity formula and position formula using new inertia weight.

(8) $$\begin{array}{c} V_{l}\left(t+1\right)=\omega \left(t\right)V_{l}\left(t\right)+c_{1}R_{1l}\left(p{\text{best}}_{l}\left(t\right)-X_{l}\left(t\right)\right)+c_{2}R_{2l}\left(\text{gbest}\left(t\right)-X_{l}\left(t\right)\right)X_{l}\left(t+1\right)=X_{l}\left(t\right)⨁V_{l}\left(t\right). \end{array}$$

The random value *R* is specified as a matrix to boost the randomness of particle swarm optimization. The random matrix of each particle is initialized with each iteration. Therefore, a group represents multiple candidate clustering centers of the data vector. Each data vector belongs to a cluster according to its membership function, so each data vector is given a fuzzy membership. In each iteration, each cluster has a cluster center, and a solution method of cluster center vector is given. The fitness function for finding the generalized solution is expressed as:

(9) $$\begin{array}{c} f\left(X_{l}\right)=\frac{1}{J\left(X_{l}\right)}. \end{array}$$

After the initial centroid is randomly selected in the traditional *K*-means clustering algorithm, the clustering results fluctuate greatly and the accuracy is low. The improved clustering proposed in this paper can optimize the initial centroid selection of the *K*-means clustering algorithm. The algorithm improves from the quantum revolving gate and changes the mutation strategy from the traditional nongate to the H gate. The improvement of the quantum revolving gate is to organically combine the three behaviors of foraging, clustering, and tail chasing in the fish school, and dynamically update the rotation angle with the increase of the number of iterations, so as to make the update of the next generation more reasonable. The algorithm, on the other hand, will run out of memory as the amount of data grows. As a result, we must concentrate on how to solve such problems using the distributed computing architecture in order to increase the algorithm's performance. The flow of the improved fuzzy clustering algorithm is shown in Figure 5.

## 4. Experiments and Results

This study adopts the methods of literature research, in-depth interview, investigation, and statistical analysis. The respondents of the questionnaire include 30 functional departments such as the academic affairs office, personnel office, science, and technology office, and student office of four vocational colleges: Nanjing Information Vocational and Technical College, Wuxi Vocational and Technical College, Yangzhou Industrial Vocational and Technical College and Changzhou Engineering Vocational and Technical College, with 300 student representatives. A total of 800 questionnaires were distributed to faculty and students of functional departments, and 750 questionnaires were recovered, of which 725 were valid, with an effective rate of 90%. However, the government's support for vocational colleges in terms of relevant policies and the coverage of special construction indicators needs to be improved, and the investment and support in the construction of high-level professional clusters and the integrated practice platform of industry education integration need to be strengthened. The analysis table of output factors of high-level scientific research projects and achievements is shown in Table 1 and Figure 6.

From the data analysis, the reason for the small number of high-level scientific research projects and achievements in some Jiangsu vocational colleges is that the mechanism and platform of collaborative innovation need to be improved, the innovation ability of scientific researchers and teams needs to be improved, and the effective allocation of scientific research resources needs to be strengthened. Therefore, the output of high-level scientific research papers and patents is still relatively rare. At the same time, it faces difficulties in the integration of industry and education and in-depth school-enterprise cooperation. It also needs to be strengthened in the service of scientific research achievements to local economic and social development. The output of scientific research projects and achievements is an important quantitative index for the development of higher vocational education, and high-level projects and achievements are the key symbols of the scientific research level of the school. The factor analysis of high-end team construction is shown in Table 2 and Figure 7.

According to the data analysis, the reason why some high-level and high-end teachers in Jiangsu vocational colleges are weak is that the proportion of highly educated teachers and professors in the teaching team of vocational colleges is relatively weak, and the level of double qualified teachers with rich enterprise experience needs to be improved. Therefore, from the perspective of supply and demand, how strengthening the introduction of high-level talents and teams and cultivating high-level technical talents will become an important problem faced by high-level vocational colleges in Jiangsu Province. The factors affecting the education and teaching quality of some Jiangsu vocational colleges include the quality of students, professional construction, and talent training quality. The construction of professional and high-level teaching achievements is the key to promoting the high-level construction of Jiangsu. Nowadays, the professional construction of Jiangsu vocational colleges still does not break the technical barriers of majors. Only by integrating the advantages of existing majors and developing cross-new disciplines can we play the role of complementary advantages among majors and promote the development and construction of majors. At the same time, the high-level teaching achievements and awards need to be enhanced.

## 5. Conclusion

Industrial college is the most important carrier for vocational colleges to realize the integration of industry and education. It is also the base for cultivating high-quality skilled applied talents. To accelerate the construction of industrial colleges, we must establish a construction mechanism and action plan that will deepen the development path of vocational colleges' integration of industry and education, implement the innovative development concept, promote higher vocational industrial colleges to better serve the new mode of vocational colleges, enterprises, and industrial cooperation in running schools, and assist vocational colleges in achieving long-term success. This paper analyzes the problems existing in the construction of industrial colleges in vocational colleges in China and finds out the corresponding solutions. A path method of industrial college construction in vocational colleges based on the cluster analysis algorithm is proposed.

The construction of the higher vocational industrial college also needs the joint efforts of the government, administration, schools, and enterprises. Only by deepening the reform of vocational education and improving the joint school running mode of multiple subjects can we achieve the two-way balance between supply and demand of talent training. We must emphasize the role of vocational education in industrial development, as well as the complimentary, balanced, and constraining link between the two. Throughout the entire process of running the Institute of Industry, the management idea of deep integration of industry and education, as well as collaborative innovation and development, will be applied. The Institute of Industry and Technology will exchange and integrate educational resources while also spearheading discipline and specialization construction reform. We also need to promote the goal of talent-oriented training, establish a stable professional teaching team, build a systematic standardized practical teaching site, and strengthen the function of school-enterprise coordinated development of industrial colleges.

## Figures and Tables

**Figure 1:** The construction path of industrial college in vocational colleges.

**Figure 2:** The development status of the Institute of Technology.

**Figure 3:** The construction path of the industrial college.

**Figure 4:** The general steps of clustering.

**Figure 5:** The flow of the improved fuzzy clustering algorithm.

**Figure 6:** Analysis on output factors of high-level scientific research projects.

**Figure 7:** Analysis on factors of high-end team construction.

**Table 1:** Analysis on output factors of high-level scientific research projects.

Project	NIVTC	WVTC	YITC	CEVTC
Innovation mechanism	12.30%	14.30%	13.50%	15.60%
Innovation platform	15.50%	12.30%	14.30%	15.30%
Teaching staff	29.80%	23.20%	22.50%	24.30%
Resource allocation	18.80%	19.20%	17.30%	16.30%
Cooperation ability	15.90%	16.20%	18.60%	18.20%
Transformation level	07.70%	14.80%	13.80%	10.30%

**Table 2:** Analysis on factors of high-end team construction.

Project	NIVTC	WVTC	YITC	CEVTC
Highly educated teachers	22.30%	20.30%	23.40%	21.60%
High-level talents	32.50%	32.10%	34.10%	35.50%
High-level team	26.80%	23.40%	22.70%	25.30%
Cultivation strength	18.40%	24.20%	19.80%	17.60%

## Data Availability

The data sets used during the current study are available from the corresponding author on reasonable request.
